# Effect of Unilateral Knee Extension Restriction on the Lumbar Region during Gait

**DOI:** 10.1155/2022/1151753

**Published:** 2022-08-22

**Authors:** Shintaro Nakatsuji, Masayuki Kawada, Yasufumi Takeshita, Yuta Matsuzawa, Kazutaka Hata, Sota Araki, Ryoji Kiyama

**Affiliations:** ^1^Doctoral Program, Division of Health Sciences, Graduate School of Health Sciences, Kagoshima University, 8-35-1 Sakuragaoka, Kagoshima City, Kagoshima 890-8544, Japan; ^2^Miyakonojo Rehabilitation Academy, 5822-9 Oiwada-cho, Miyakonojo City, Miyazaki 885-0062, Japan; ^3^Department of Physical Therapy, School of Health Sciences, Faculty of Medicine, Kagoshima University, 8-35-1 Sakuragaoka, Kagoshima City, Kagoshima 890-8544, Japan

## Abstract

Unilateral knee extension restriction might change trunk alignment and increase mechanical load on the lumbar region during walking. We aimed to clarify lumbar region mechanical load during walking with restricted knee extension using a musculoskeletal model simulation. Seventeen healthy adult males were enrolled in this study. Participants walked 10 m at a comfortable velocity with and without restricted right knee extension of 15° and 30° using a knee brace. L4–5 joint moment, joint reaction force, and muscle forces around the lumbar region during walking were calculated for each condition. Peaks of kinetic data were compared among three gait conditions during 0%–30% and 50%–80% of the right gait cycle. Lumbar extension moment at early stance of the bilateral lower limbs was significantly increased in the 30° restricted condition (*p* < 0.001). Muscle force of the multifidus showed peaks at stance phase of the contralateral side during walking, and the erector spinae showed force peaks at early stance of the bilateral lower limb. Muscle force of the multifidus and erector spinae increased with increasing degree of knee flexion (*p* ≤ 0.010), with a large effect size (*η*^2^ = 0.273–0.486). The joint force acting on L4–5 showed two peaks at early stance of the bilateral lower limbs during the walking cycle. The anterior and vertical joint force on L4–5 increased by 14.2%–36.5% and 10.0%–23.0% in walking with restricted knee extension, respectively (*p* ≤ 0.010), with a large effect size (*η*^2^ = 0.149–0.425). Restricted knee joint extension changed trunk alignment and increased the muscle force and the vertical and anterior joint force on the L4–5 joint during walking; this tendency became more obvious with increased restriction angle. Our results provide important information for therapists engaged in the rehabilitation of patients with knee contracture.

## 1. Introduction

Increased musculoskeletal stress repeated during daily activities leads to pain or movement disorders. Thus, knowledge of the load on joints and muscles during daily activity and exercise is useful information for understanding the clinical condition of patients and planning an appropriate therapeutic program during musculoskeletal rehabilitation. Dysfunction of the lower limbs affects the kinematics and kinetics of the entire body during stance.

Knee joint plays an important role during walking. It supports the body weight in the stance phase and adjusts the lower limb length by changing the relative angle between the lower leg and thigh in the swing phase [1]. These knee functions contribute to efficient and safe walking. Unilateral restriction of knee extension caused by knee osteoarthritis or orthopaedic surgery increases posterior tilt, lateral tilt to the affected side of the pelvis, lumbar kyphosis, and lateral tilt of the trunk in the standing position [2–6]. During walking, unilateral restriction of knee extension also changes the gait kinematics as follows: it increases anterior tilt of the pelvis and trunk, and increases lateral tilt towards the unaffected side during the stance phase [7]. These changes in the postural alignment of the entire body are associated with low back pain. A previous study reported that 58.1% of patients with knee osteoarthritis have low back pain [8]; this relationship between knee dysfunction and low back pain is called knee-spine syndrome [9, 10].

Kinetic changes during walking with a restricted extension of the knee joint have been analysed in previous studies where knee joint force was bilaterally increased during loading response depending on the degree of restriction of the knee joint [11–13]. Knee extension restriction also increases the vertical component of ground reaction force and the external knee flexion moment, which increases the demand for muscle activity in the lower extremities [14–17]. Gait kinematics and kinetics due to restriction of knee extension might increase the load on the lumbar region during the loading response phase of the restricted lower limb during gait and is related to low back pain. Although knowledge regarding a change in the lumbar load during walking, caused by the restriction of knee extension, is necessary for therapists engaged in the rehabilitation of patients with knee injuries, there is a dearth of studies that have analysed this issue.

Lumbar load during gait is usually analysed by muscle activity measured using electromyography. Various studies report that increased trunk sway increases the stress on lumbar muscles during gait [18–21]. However, action potential obtained from electromyography correlates with muscle force only in isometric contractions, but not in concentric and eccentric contractions. Thus, the muscle action potential does not necessarily reflect the mechanical stress of the muscle. These issues make it difficult to analyse lumbar load during movement.

Meanwhile, musculoskeletal model simulation becomes useful for estimating the muscle force of whole-body muscles in human movement science. A musculoskeletal model simulation can noninvasively quantify the joint load, based on inverse dynamics and an optimization method from the kinematic data obtained by motion capture [22–26]. Musculoskeletal model simulation can estimate both joint force and muscle force. In other words, a musculoskeletal model simulation contributes to our understanding of the relationship between load on muscle and joints and kinematic human movement.

To date, the mechanical load on the lumbar region during walking with unilateral restricted knee extension has not been clarified due to a lack of studies employing musculoskeletal model simulation. The purpose of this study is to clarify the mechanical load on the lumbar region during walking with restricted knee extension, comparing the load during normal walking, using musculoskeletal model simulation. Mechanical load on the lumbar region was estimated by the lumbar muscle force, internal joint moment, and joint force on L4–5. We hypothesized that unilateral restriction of knee extension increased the mechanical load of the lumbar region at the ipsilateral stance phase during walking, and this tendency would be more obvious as restriction of the knee angle increased.

## 2. Materials and Methods

### 2.1. Participants

Seventeen healthy adult males with no orthopaedic or neurological disorders influencing normal gait in the lumbar region and lower limbs (age, 26.0 ± 2.2 y; height, 1.69 ± 0.05 m; weight, 62.5 ± 5.6 kg; average ± standard deviation; 16 right footed and 1 left footed) participated in this study. The Medical clearance was preliminarily obtained by a physical therapist's interview. The participants were given a written and oral explanation of the purpose and content of the study, and their consent was obtained in writing in accordance with the principles stipulated in the Declaration of Helsinki. Participants were advised that participation in the research was voluntary and they would incur no disadvantage even if they decided not to participate in the research or withdrew their consent. This study was approved by the Ethics Committee on Epidemiology and Clinical Research of the Faculty of Medicine, Kagoshima University (number, 180095Epi ver2).

### 2.2. Measurement and Procedures

A motion analysis system consisting of eight infrared cameras was used to measure gait with and without restricted extension of the right knee joint. The sampling frequency was 100 Hz for the infrared camera. Retroreflective markers were placed in accordance with the plug-in-gait model; we also placed markers on the medial epicondyle and medial malleolus, and plates with three reflex markers on the bilateral thigh and shank [27, 28]. Right knee extension was restricted by 15° and 30° using a knee brace with bilateral struts [6, 7, 29]. Flexion of the right knee joint was not restricted. First, we confirmed whether the maximum knee extension angle during walking was restricted as intended. Participants randomly performed 10-m walking with and without a restricted knee joint at a comfortable speed five times after several rounds of practice in each gait condition.

The noise was removed from the kinematic data measured by the motion capture system using a Butterworth low-pass filter with a cut-off frequency of 6 Hz. Then, the kinematic data were input to the musculoskeletal model (AnyBody 7.1, AnyBody Technology, Aalborg, Denmark). The internal joint moment, muscle force, and joint reaction force around the lumbar region during walking were estimated by musculoskeletal model simulation. The effect of the extension limitation of the right knee joint on the mechanical load of joints and muscles around the lumbar region was analysed.

The MoCap full-body model of the AnyBody Managed Model Repository v.2.1.1 was used as the musculoskeletal model. The degrees of freedom of this model were 42, and the L4–5 intradiscal joint was defined as a joint with 3 degrees of freedom. For the muscle contraction model, we used a Hill-type model that considered characteristics such as parallel contraction elements and passive elements of muscles, in-line tendon elasticity, and pinnate angle of muscle fibres [30].

The ground reaction force was also estimated by the optimization method for further kinetic analysis. Twenty-four points of contact with the floor were defined on the bilateral sole of the musculoskeletal model, and the presence or the absence of contact was determined by the distance to the floor and the relative acceleration [31]. The ground reaction force was estimated so that it balanced the sum of the mass-acceleration product of all body segments and the gravity acting on the whole body [32]. Then, the joint moment, joint reaction force, and muscle force around the lumbar region during walking were calculated using inverse dynamics and optimization methods. Optimization was performed to minimize the sum of the cubes of the muscle load expressed by the ratio of the exerted muscle output to the maximum muscle strength of each muscle [33]. The muscle force of the bilateral lumbar multifidus and erector spinae was calculated. The muscle force of the erector spinae and iliocostalis muscles was calculated as the sum of forces generated by those fibres crossing L4–5. The joint reaction force acting on L4 from L5 was estimated based on the local coordinate system of L5, referring to the recommendation by the International Society of Biomechanics [34, 35]. We initially examined the validity of the joint moment, the joint reaction force of L4–5, and the muscle force of the lumbar region estimated by predicted ground reaction force compared with those calculated using measured ground reaction force. The values obtained from the two methods were very similar, and intraclass correlation coefficients _(2,1)_ were very high, 0.97–1.00 (95% confidence level, 0.87–1.00; *p* < 0.001).

Trunk angle was defined as the angle of the thorax segment relative to the global coordinate system. Thorax coordinate system was defined by the makers attached to the jugular incision, xiphoid process, and spinous process of the C7 vertebra and T8 vertebra, according to the recommendation by International Society of Biomechanics [36]. The walking speed and walking cycle were calculated from the trajectory of the markers on both heels. Time of the kinematic and kinetic data was normalized as 100% for the right walking cycle duration; joint moment, joint reaction force, and muscle force were also normalized by body weight. The waveforms for five trials were averaged to produce an ensemble average waveform for each participant.

### 2.3. Statistical Analysis

Peak values of kinematic and kinetic data of the sagittal and frontal planes were compared among three gait conditions during 0%–30% and 50%–80% of the right gait cycle, according to a previous study [19]. These analysis sections correspond to the early stance and early mid-stance phases of both lower limbs. Trunk angle, joint moment, muscle force, and joint reaction force were compared to examine the effect of unilateral knee extension restriction on the mechanical lumbar load. The normality of data distribution was confirmed by the Shapiro–Wilk test. Repeated-measures analysis of variance (ANOVA) was performed if the normal distribution was able to be assumed, or Friedman test was performed in cases where normal distribution could not be assumed. Tukey's test or Wilcoxon's rank-sum test with Bonferroni correction was used as post hoc tests. Meanwhile, *η*^2^ was calculated to estimate the effect size in ANOVA and the Friedman test. Effect size was classified into small (*η*^2^ = 0.01), medium (*η*^2^ = 0.06), and large (*η*^2^ > 0.14), according to a previous study [37]. SPSS Statistics 26.0 was used as the statistical software, and the threshold of significance was established at 0.05.

## 3. Results

Gait velocities under 15° and 30° restricted knee conditions were 0.88 ± 0.18 m/s and 0.86 ± 0.18 m/s, respectively, showing a significantly slower velocity than normal walking of 1.11 ± 0.11 m/s (Table 1). The maximum right knee extension angle was -4.2 ± 4.9° during normal walking, -17.0 ± 7.7° in the 15° restricted condition, and -27.3 ± 0.2° in the 30° restricted condition, respectively (Table 1). Similarly, a decreased knee extension angle was also observed in the left knee joint of the unrestricted side. Trunk flexion angle throughout a gait cycle was increased with an increment in knee restriction angle (Figure 1(a); Table 1).

L4–5 moment showed peaks during early stance of the bilateral lower limb. Lumbar extension moment at the early stance of the restricted side was significantly increased by 1.7- and 2.2-fold under the 15° and 30° restricted conditions compared with normal walking, respectively (Figure 1(c); Table 2). The difference in L4–5 extension moment of the restricted side had a large effect size (*η*^2^ = 0.543). Lumbar extension moment at early stance of the unrestricted side showed similar results. The lateral lumbar moment to the right, in the 30° restriction condition, was significantly increased compared to that during normal walking at the early stance of the unrestricted side (Figure 1(d); Table 2).

Muscle force of the multifidus showed peaks at the stance phase of the contralateral side during walking, and the erector spinae showed force peaks at early stance of the bilateral lower limb (Figure 2). Muscle force of the right multifidus at early stance of the unrestricted side was significantly increased to 3.3- and 4.3-fold compared with normal gait by the 15° and 30° restriction of the right knee joint, respectively (Figure 2(a); Table 2). Muscle force at early stance of the left multifidus significantly increased muscle force to 2.3- and 3.3-fold of those during normal gait. Similarly, the right erector spinae significantly increased peak force by 28.0% and 54.5% at early stance of the restricted lower limb, and 68.1% and 101.7% at early stance of the unrestricted lower limb due to the 15° and 30° restricted conditions (Figure 2(b); Table 2). The left erector spinae showed similar results to the right erector spinae (Figure 2(b); Table 2). The difference in muscle force of the multifidus and erector spinae had a large effect size (*η*^2^ = 0.273–0.486).

A joint force acting on L4–5 showed two peaks at early stance of the bilateral lower limb during the walking cycle (Figure 3). The anterior force of L4–5 at early stance of the unrestricted lower limb was significantly increased by 25.3% in the 15° restricted condition and 36.5% in the 30° restricted condition compared with normal walking (Figure 3(a); Table 2). Vertical force of L4–5 during gait with the 30° restricted knee increased significantly by 10.0% at early stance of the restricted lower limb, and 23.0% at early stance of the unrestricted lower limb compared with normal walking, respectively (Figure 3(c); Table 2). Differences in the anterior and vertical forces of L4–5 had a large effect size (*η*^2^ = 0.149–0.425).

## 4. Discussion

This is the first study that verified mechanical load on muscles and joints of the lumbar region during walking with unilateral knee extension restriction to our knowledge. Consistent with our hypothesis, the current results showed that the muscle force and joint reaction force of the lumbar region were increased as the degree of knee restriction increased. Meanwhile, increased load on the lumbar region was unexpectedly observed in the stance phase of the bilateral lower limb. These findings are important information for therapists engaged in the rehabilitation of patients with knee contracture to prevent the secondary disorders such as low back pain.

The extension moment between L4 and L5 was 0.15–0.17 Nm/kg during normal walking in this study, adding support to previous studies [19, 20, 38]. Restricted knee joint extension increased mechanical load on the lumbar region during walking, despite the decrease in walking speed. Restricted knee extension increased the lumbar extension and right flexion moment compared with normal walking. In particular, the increase in extension moment was large, increasing by 70.6%–123.5% at the 15° restriction and 126.7%–193.3% at the 30° restriction condition compared with normal walking. Trunk alignment alteration due to restriction of the knee joint would have increased the lumbar extension moment. Similar to previous findings [6, 7], right knee restriction during walking increased trunk flexion and right flexion angle during gait. Restriction of knee extension increased the distance between the ground reaction force vector and the centre of the knee joint of early stance of the restricted side during walking, resulting in an increase in internal knee joint extension moment. Forward tilt of the trunk would occur to suppress an increase in the knee joint extension moment, caused by a forward shift of the mass of the upper body and reduced moment arm of the ground reaction force around the knee joint. On the other hand, the forward tilt of the trunk increased the moment arm of the ground reaction force around the L4–5 joint, resulting in an increase in L4–5 extension moments. In addition, the difference of lower limb length, owing to the restricted knee joint, increased trunk lateral inclination to the restricted side, resulting in increased L4–5 right flexion moment.

Increased lumbar extension moment was observed also at early stance of the unrestricted lower limb. Maximal extension angle of the left knee (the unrestricted side) was decreased similarly to the restricted knee joint during walking. Unilateral restriction of the knee joint caused a difference in bilateral leg length, resulting in asymmetry of pelvis and trunk motion during gait. Participants with unilateral restriction of knee extension walked with an optional flexed knee joint to suppress the asymmetrical trunk movement. On the other hand, this gait alteration increased the bilateral knee extensor muscle load. Thus, compensation through a forward trunk tilt was also observed during stance phase of the contralateral lower limb, and an increased L4–5 extension moment appeared similarly in the stance phase of the restricted side. Those increased lumbar moment required greater muscle force of the bilateral multifidus and erector spinae than during normal walking.

The vertical and anterior components of the joint force on L4–5 in normal walking were at a maximum between the loading response phase and the mid-stance phase, approximately 117%–130% body weight (BW) and 15%–17% BW in this study, respectively. Similarly, in a previous study [39] that analysed the joint force on L4–5 during walking, calculated using a musculoskeletal model, the vertical component was the largest at 20% and 60% of the gait cycle, and the value was 102%–128% BW. In the current study, the anterior and vertical joint force on L4–5 increased by 14.2%–36.5% and 10.0%–23.0% in walking with restricted knee extension, respectively. Increased muscle force of the multifidus and erector spinae generates a compressive force acting on L4–5 vertebral bodies and increases the joint force. Increased forward tilt of the trunk also imposes an effect of gravity during action on the L4–5 joint surface; thus, the anterior component of the joint force was increased [40].

In this study, we have demonstrated that restricted knee joint extension changed trunk alignment and increased the muscle force of the multifidus and erector spinae and the vertical and anterior joint force on the L4–5 joint during walking; this tendency became more obvious as the restriction angle was increased. The compressive and anterior forces created might increase the load on adjacent vertebrae, and shear force on the facet joints. Unexpectedly, a twice increased load was observed during one walking cycle in the erector. Walking is a repetitive motion during daily life; therefore, repetitive stress that can accumulate on muscles and lumbar joints might trigger low back pain [41–43].

Our study had a limitation related to the participants. We analysed simulated walking with restriction on knee extension; therefore, gait adaptation might be different from that in patients with restriction on knee extension owing to osteoarthritis. However, trunk forward tilt is usually observed during gait adaptation in patients with knee osteoarthritis in a similar manner to the results of this study. We also analysed small sample size for young male subjects in this study; therefore, careful consideration is needed to apply our results to females and older people. Future studies are needed to clarify the effect of restricted knee extension on the lumbar region load in various people, including patients with knee osteoarthritis.

## 5. Conclusions

The present study demonstrates that unilateral knee extension restriction changed trunk alignment and increased the mechanical load of the lumbar region during walking. These findings supported our hypothesis that the mechanical load became more pronounced as the angle of knee restriction increased. Our results provide important information for therapists engaged in the rehabilitation of patients with knee contracture.

## Figures and Tables

**Figure 1:** The ensemble average of all participants of sagittal trunk motion (a) lateral trunk motion (b) sagittal L4–5 internal joint moment (c) and lateral L4–5 internal joint moment (d) “Normal” denotes normal walking, and “15°” and “30°” indicate the condition concerning the right knee extension restriction. Time was normalized across the whole gait cycle of the right lower limb. The shaded regions indicate early stance of the bilateral lower limbs and peaks that were analysed statistically. ^*∗*^ and ^*∗∗*^indicate a significant difference between the normal condition at *p* < 0.05 and *p* < 0.01, respectively. † and ‡ indicate significant difference between 15° at *p* < 0.05 and *p* < 0.01, respectively.

**Figure 2:** The ensemble average of all participants of the bilateral multifidus (a) and erector spinae (b) “Normal” denotes normal walking, and “15°” and “30°” indicate the right knee extension restriction condition. Time was normalized across the whole gait cycle of the right lower limb. The shaded regions indicate early stance of the bilateral lower limbs, and peaks of those were analysed statistically. ^*∗*^ and ^*∗∗*^indicate a significant difference between the normal condition at *p* < 0.05 and *p* < 0.01, respectively. † and ‡ show significant difference between 15° at *p* < 0.05 and *p* < 0.01, respectively.

**Figure 3:** The ensemble average of all participants of anterior force (a) lateral force (b) and vertical force (c) acting on the L4–5 joint. “Normal” denotes normal walking, and “15°” and “30°” indicate the right knee extension restriction condition. Time was normalized across the whole gait cycle of the right lower limb. The shaded regions indicate early stance of the bilateral lower limbs, and peaks of those were analysed statistically. ^*∗*^ and ^*∗∗*^indicate a significant difference between the normal condition at *p* < 0.05 and *p* < 0.01, respectively. † shows the significant difference of 15° at *p* < 0.05.

**Table 1:** Gait velocity, knee, and trunk angle during gait under three conditions (mean ± standard deviation).

		Normal	15°	30°	*F* or *χ*^2^	*p* value	*η* ^2^
Gait velocity (m/s)		1.11 ± 0.11	0.88 ± 0.18^*∗∗*^	0.86 ± 0.18^*∗∗*^	*F* = 30.49	<0.001	0.337
Right knee extension							
Angle (°)		−4.2 ± 4.9	−17.0 ± 7.7^*∗*^	−27.3 ± 0.2^*∗∗*^†	*χ* ^2^ = 34.00	<0.001	1.000
Moment (Nm/kg)		0.51 ± 0.24	0.73 ± 0.28^*∗*^	0.86 ± 0.37^*∗∗*^	*χ* ^2^ = 17.29	<0.001	0.509
Left knee extension							
Angle (°)		−4.9 ± 5.6	−12.3 ± 7.7^*∗∗*^	−17.1 ± 9.7^*∗∗*^†	*F* = 24.14	<0.001	0.290
Moment (Nm/kg)		0.55 ± 0.22	0.57 ± 0.29	0.69 ± 0.33†	*F* = 4.06	0.027	0.043
Trunk angle (°)							

Flexion	1st	−4.9 ± 3.7	−11.1 ± 6.1^*∗∗*^	−14.6 ± 6.8^*∗∗*^‡	*F* = 23.77	<0.001	0.345
	2nd	−4.5 ± 3.5	−11.5 ± 6.5^*∗∗*^	−14.8 ± 7.0^*∗∗*^†	*F* = 26.09	<0.001	0.363

Lateral	1st	1.6 ± 2.2	2.4 ± 2.3	3.2 ± 2.7^*∗∗*^	*χ* ^2^ = 10.42	0.005	0.306
	2nd	−0.4 ± 2.2	−1.2 ± 2.7	−0.8 ± 3.3	*F* = 1.39	0.263	0.013

1st indicates the peak of 0%–30%, and 2nd indicates the peak of 50%–80% of the right gait cycle. ^*∗*^*p* < 0.05 vs. Normal; ^*∗∗*^*p* < 0.01 vs. Normal; †*p* < 0.05 vs. 15; ‡*p* < 0.01 vs. 15°.

**Table 2:** Internal joint moment, muscle force, and joint force around the L4–5 joint during gait under three conditions (mean ± standard deviation).

		Normal	15°	30°	*F* or *χ*^2^	*p* value	*η* ^2^
L4–5 moment (Nm/kg)							
Extension	1st	0.17 ± 0.08	0.29 ± 0.11	0.38 ± 0.15^*∗*∗†^	*χ* ^2^ = 18.47	<0.001	0.543
	2nd	0.15 ± 0.08	0.34 ± 0.15^*∗∗*^	0.44 ± 0.16^*∗*∗‡^	*F* = 29.30	<0.001	0.440
Lateral	1st	−0.20 ± 0.04	−0.24 ± 0.06	−0.24 ± 0.07	*F* = 4.38	0.021	0.093
	2nd	0.18 ± 0.06	0.22 ± 0.06	0.24 ± 0.08^*∗*^	*F* = 7.55	0.002	0.120

Muscle force (%BW)							
Multifidus	Right	1.64 ± 1.12	5.42 ± 2.71^*∗∗*^	7.03 ± 3.38^*∗∗*^	*F* = 28.81	<0.001	0.433
	Left	1.57 ± 0.80	3.65 ± 1.94^*∗∗*^	5.25 ± 2.32^*∗*∗‡^	*F* = 27.32	<0.001	0.411

Erector spinae							
Right	1st	20.49 ± 12.25	26.22 ± 12.05	31.66 ± 8.77^*∗*^	*χ* ^2^ = 9.29	0.010	0.273
	2nd	21.55 ± 7.84	36.23 ± 11.80^*∗∗*^	43.47 ± 12.75^*∗*∗†^	*F* = 22.67	<0.001	0.407
Left	1st	23.88 ± 10.08	33.06 ± 13.17	40.49 ± 14.14^*∗*∗†^	*χ* ^2^ = 15.65	<0.001	0.460
	2nd	15.50 ± 5.79	29.85 ± 10.24^*∗∗*^	36.33 ± 10.10^*∗*∗†^	*F* = 26.42	<0.001	0.486

L4–5 force (%BW)							
Anterior	1st	17.45 ± 10.88	18.23 ± 10.16	19.93 ± 5.55	*χ* ^2^ = 5.06	0.080	0.149
	2nd	15.03 ± 3.82	18.83 ± 3.96^*∗*^	20.52 ± 3.30^*∗∗*^	*F* = 12.34	<0.001	0.425
Lateral	1st	2.18 ± 0.94	1.87 ± 1.15	1.86 ± 1.27	*F* = 2.32	0.115	0.017
	2nd	−2.08 ± 0.53	−1.93 ± 1.03	−1.97 ± 1.11	*F* = 0.22	0.800	0.004
Vertical	1st	130.23 ± 74.79	136.87 ± 69.58	143.27 ± 34.21^†^	*χ* ^2^ = 9.29	0.010	0.273
	2nd	117.46 ± 18.43	133.43 ± 23.70	144.49 ± 21.16^*∗*^	*F* = 7.50	0.002	0.204

1st indicates the peak of 0%–30%, and 2nd indicates the peak of 50%–80% of the right gait cycle. ^*∗*^*p* < 0.05 vs. Normal; ^*∗∗*^*p* < 0.01 vs. Normal; †*p* < 0.05 vs. 15°; ‡*p* < 0.01 vs. 15°.

## Data Availability

The data used to support the findings of the current study can be obtained from the corresponding author upon request.
